RETRACTED

# Establishment and Evaluation of Artificial Intelligence-Based Prediction Models for Chronic Kidney Disease under the Background of Big Data

**DOI:** 10.1155/2022/6561721

**Published:** 2022-07-08

**Authors:** Xiaoqian Yan, Ximin Li, Ying Lu, Dongfang Ma, Shenghong Mou, Zhiyuan Cheng, Yuan Ding, Bin Yan, Xianzhen Zhang, Gang Hu

**Affiliations:** ^1^Department of Nephropathy, Tongde Hospital of Zhejiang Province, Hangzhou, Zhejiang 310012, China; ^2^School of Micro-Nanoelectronics, Zhejiang University, Hangzhou, Zhejiang 310058, China; ^3^Network Information Center, Tongde Hospital of Zhejiang Province, Hangzhou, Zhejiang 310012, China

## Abstract

**Objective:**

To establish a prediction model for the risk evaluation of chronic kidney disease (CKD) to guide the management and prevention of CKD.

**Methods:**

A total of 1263 patients with CKD and 1948 patients without CKD admitted to the Tongde Hospital of the Zhejiang Province from January 1, 2008, to December 31, 2018, were retrospectively analyzed. Spearman's correlation was used to analyze the relationship between CKD and laboratory parameters. XGBoost, random forest, Naive Bayes, support vector machine, and multivariate logistic regression algorithms were employed to establish prediction models for the risk evaluation of CKD. The accuracy, precision, recall, F1 score, and area under the receiver operating curve (AUC) of each model were compared. The new bidirectional encoder representations from transformers with light gradient boosting machine (MD-BERT-LGBM) model was used to process the unstructured data and transform it into researchable unstructured vectors, and the AUC was compared before and after processing.

**Results:**

Differences in laboratory parameters between CKD and non-CKD patients were observed. The neutrophil ratio and white blood cell count were significantly associated with the occurrence of CKD. The XGBoost model demonstrated the best prediction effect (accuracy = 0.9088, precision = 0.9175, recall = 0.8244, F1 score = 0.8868, AUC = 0.8244), followed by the random forest model (accuracy = 0.9020, precision = 0.9318, recall = 0.7905, F1 score = 0.581, AUC = 0.9519). Comparatively, the predictions of the Naive Bayes and support vector machine models were inferior to those of the logistic regression model. The AUC of all models was improved to some extent after processing using the new MD-BERT-LGBM model.

**Conclusion:**

The new MD-BERT-LGBM model with the inclusion of unstructured data has contributed to the higher accuracy, sensitivity, and specificity of the prediction models. Clinical features such as age, gender, urinary white blood cells, urinary red blood cells, thrombin time, serum creatinine, and total cholesterol were associated with CKD incidence.

RETRACTED

## 1. Introduction

Chronic kidney disease (CKD) is a major disease with high morbidity and mortality. It imposes a large economic burden on the patients, healthcare system, and society. Its early clinical manifestations are not obvious and are thus often overlooked by patients or even general practitioners, leading to some patients missing the best timing for treatment. Among the population aged over 20 years old in high-income countries, the prevalence of CKD is approximately 8.6% in men and 9.6% in women [1]. Patients with CKD have a shorter life expectancy than the general population due to their increased risk of cardiovascular disease [2]. CKD and its comorbidities are also important drivers of health care costs. Fortunately, timely treatment can effectively control the progression of CKD and even prevent it [3].

Nephrologists and researchers have been striving relentlessly to develop new strategies for the early diagnosis of CKD so as to delay its progression and prevent one of its final outcomes, that is renal failure, because CKD can be prevented by early diagnosis and appropriate therapy. Further, timely treatment of its comorbidities such as diabetes, obesity, and hypertension is also key to the primary prevention of CKD. Secondary prevention of CKD depends on screening and accurately identifying high-risk groups, which could contribute to early detection and treatment [4]. In the current literature, the limitations of existing studies related to the risk assessment of CKD revolve around a limited number of laboratory tests. In addition, the pathogenesis of CKD is complex and multifactorial, making it difficult to simply explain in a linear relationship.

Artificial intelligence (AI) is an interdisciplinary discipline that has attracted much attention, with unique learning techniques to simulate human intelligence [5, 6]. AI adapts to the diversity of data through algorithms and can compensate for the shortcomings of analyzing CKD risks. Therefore, this study established an AI prediction model to evaluate the risk of CKD. With the cooperation of clinicians and computer engineers, a large amount of real-world electronic medical records were collected for AI analysis, which were then validated.

## 2. Methods and Materials

### 2.1. Source of Data

A total of 30,231 cases hospitalized in the Department of Internal Medicine at the Tongde Hospital of Zhejiang Province (Zhejiang, China) from January 1, 2008, to December 31, 2018, were retrospectively analyzed and converted into computer-readable data. They were divided into CKD and non-CKD groups based on the 2002 Kidney Disease Improving Global Outcomes diagnosis criteria for CKD [7]. After excluding cases with a follow-up time of less than 3 months and those with missing laboratory data that could not determine the presence of CKD, 1902 CKD cases and 21,832 non-CKD cases were obtained. Finally, 1263 CKD cases and 1948 non-CKD cases were collected after excluding cases with significant data loss. The medical records of all study subjects were then collected during admission, including age, gender, and laboratory indicators in blood and urine. All patients provided informed consent. This study was approved by the Medical Ethics Committee of Tongde Hospital of the Zhejiang Province (YJSKTSC2019001).

RETRACTED

### 2.2. Modeling and Analysis

The data of all study subjects were integrated and divided into a training set and a test set in a 9 : 1 ratio. XGBoost, random forest (RF), Naive Bayes (NB), support vector machine (SVM), and multivariate logistic regression algorithms (LR) were used to construct models for predicting CKD risk. The accuracy, precision, recall, F1 score, and area under the receiver operating curve (AUC) of each model were compared to evaluate their predictive values. Besides, the association between the characteristic parameters in each model and the incidence of CKD was also analyzed.

To make the models closer to the real-world scenarios, this study innovatively adopted multimodal machine learning combined with Bidirectional Encoder Representations from Transformers with Light Gradient Boosting Machine (MD-BERT-LGBM). Thus unstructured data unavailable for calculation could be converted into unstructured vectors that could be calculated. Also, the medical history in the medical records was included in the model analysis to avoid missing “unknown characteristics” that could be related to the pathogenesis of CKD. The MD-BERT-LGBM model consists of six parts: (1) unstructured data, including subjects' history records and diagnosis records; (2) feature extractor, which converted unstructured data into unstructured vectors through a pretrained BERT model; (3) structured data, including demographic and laboratory test variables such as age, serum creatinine, estimated glomerular filtration rate, and urinary protein, could be directly expressed as structured vectors; (4) classification (CLS) vectors and structured data vectors directly form multimodal vectors; (5) multimodal vector training was performed, and the output could be applied to update the parameters of the trained BERT model by a backpropagation algorithm [8]; and (6) multimodal vector training of the LGBM classifier was performed, with the output indicating the risk of CKD or disease aggravation. In this study, the LGBM model was developed from the LightGBM package (version 2.3.1) [9], and the LR model from the Scikit-learn library (version 0.19.2) [10].

RETRACTED

### 2.3. Statistical Analysis

All data was statistically analyzed using the SPSS 26.0 software. Normally, distributed measurement data were expressed as mean ± standard deviation (SD), and the *t*-test was used for between-group comparison. Enumeration data were shown as frequency or percentage, and the *χ*^2^ test was used for comparison between groups. Spearman's correlation was used to analyze the correlation between CKD occurrence and laboratory test parameters. *P* < 0.05 indicated significant statistical difference.

## 3. Results

### 3.1. General Information of the Patients

A total of 1263 CKD cases and 1948 non-CKD cases were assessed. No significant difference was found in the gender ratio between the two groups. Compared with patients from the non-CKD group, patients in the CKD group were much elder and had significantly higher levels of lymphocyte/monocyte ratio, white blood cell count, urine glucose positivity, urine white blood cell positivity, urine occult blood positivity, urine white blood cells, urine red blood cells, serum potassium, total cholesterol, triglyceride, direct bilirubin, fasting blood glucose, blood urea nitrogen, serum creatinine, blood uric acid, albumin, globulin, thrombin time, and international normalized ratio, as well as a lower platelet count. Additionally, no significant difference was observed between the two groups in hemoglobin, blood sodium, low-density lipoprotein, total bilirubin, alanine aminotransferase, and fibrinogen levels (Table 1).

### 3.2. Correlation between the Occurrence of CKD and Laboratory Test Parameters

The results of Spearman correlation analysis demonstrated that neutrophil ratio, white blood cell count, red blood cell distribution width, urine red blood cells, urine occult blood, urine white blood cells, thrombin time, blood urea nitrogen, serum creatinine, blood uric acid, and globulin were positively correlated with the incidence of CKD, while red blood cell count, platelet count, and platelet distribution width were negatively correlated with the incidence of CKD (Table 2).

### 3.3. Ranking Laboratory Test Indicators Based on XG Boost Model

Based on the processing results of the data set by XGBoost, the top 15 main characteristics were ranked from high to low according to the obtained values: protein, urine red blood cells, age, serum creatinine, gender, albumin-creatinine ratio, leukocyte, erythrocyte, platelet distribution width, high-sensitivity C-reactive protein, hemoglobin, hemoglobin A1c, platelet, albumin and potassium. Notably, protein (0.220), urine red blood cells (0.209) and serum creatinine (0.032) were at the higher level of the model, while serum cholesterol and glycosylated hemoglobin were also indicators of relatively high importance for assessing the risk of CKD (Table 3).

RETRACTED

### 3.4. Comparison of the Predictive Effects of Five Models

The prediction effects of the four models were compared with those of the logistic regression model. The XGBoost model showed the highest accuracy, precision, recall, F1 score and AUC (accuracy = 0.9088, precision = 0.9175, recall = 0.8244, F1 score = 0.868, AUC = 0.8244) than the logistic regression model, with its precision and recall increased by 13.1 and 10.1 percentage points, respectively. The random forest model was the second-best model (accuracy = 0.9020, precision = 0.9318, recall = 0.7905, F1 score = 0.581, AUC = 0.9519). Except for the above two, both the Naive Bayes model and the BERT model had worse prediction performance than the logistic regression model (Table 4, Figure 1). After processing the unstructured data into researchable unstructured vectors using the new MD-BERT-LGBM model, the AUC of all models was improved to some extent compared with the traditional algorithm without unstructured data (Table 4).

## 4. Discussion

Early prediction of renal damage is vital to the prevention and treatment of CKD. A decreased glomerular filtration rate and increased urinary protein are important markers of CKD. However, when laboratory tests indicate that the glomerular filtration rate has been altered, this could suggest that the optimal timing of intervention has been missed, and impaired renal function could occur. Urine samples are a good source for assessing the severity of CKD because they contain important biomarkers suggesting the health of the kidneys. Urine markers thus serve as an effective method for detecting CKD and predicting the progression of CKD [11, 12], such as urinary kidney injury molecule-1 (KIM-1), neutrophil gelatinase-associated lipocalin (NGAL), high-mobility group box protein 1 (HMGB1), insulin-like growth factor-binding protein (IGFBP7) [13–15]. However, these markers have failed to predict whether non-CKD populations would develop CKD. Further, a single biomarker does not seem to fully describe the changes in renal function relevant to the complex pathophysiology of CKD.

One of the limitations of current electronic medical records is that the datasets often have missing and noisy values [16]. The advent of data mining has enabled a reduction in errors and improvements in data quality [17]. In this regard, using AI to mine database systems has led to efficient noise removal strategies and improved data accuracy, contributing to better learning performance and building more reliable machine learning algorithms. This is possible because deep learning models can improve machine learning algorithms by automatically computing an “abstract” interpretation of data into accurate algorithms that can be used to develop clinical decision-making models for guiding the prediction of prognosis in clinical practice [16, 17]. Thus, compared to classical mathematical models, the Al method in this study can more efficiently and accurately outline nonlinear relationships between common patient variables and accurately identify reliable variables, as illustrated in the correlation analysis of Table 2 and the ranking of the top main 15 XGBoost model features in Table 3. Further, as shown in Table 4, after the unstructured data were processed using the MD-BERT-LGBM model, improvements in the AUC of all models could be observed compared with the traditional algorithm without unstructured data, which could not be possible using traditional mathematical models. Thus, clinically, if early changes in these top main 15 indicators are observed, these could be used as a trigger for nephrologists to undertake necessary precautionary measures to prevent CKD or delay its progression by offering timely therapies to improve treatment outcomes and the patients' quality of life and survival.

RETRACTED

A meta-analysis found that serum phosphorus level was an independent risk factor for the deterioration of renal function, and each 1 mg/dl increase in serum phosphorus level was associated with an increased risk of end-stage renal failure (HR: 1.36; 95% CI, 1.20–1.55) [18]. High-protein diet, infection, hypertension, hyperlipidemia, hypercoagulable state, hypovolemia, water-electrolyte imbalance, urinary tract obstruction, nephrotoxic drug use, anemia, heart failure, obesity, and smoking have been shown to be important factors affecting the progression of CKD [19]. However, there remain some questions plaguing clinicians—whether the factors affecting CKD progression are limited to the above, how much their influence is, and whether drugs have different effects at different stages of CKD [20, 21]. These problems cannot be solved by merely large-sample regression statistical analysis. Consequently, the learning technology of AI is essential. Thus, in this present study, all metrics of easily available and commonly used specimens, blood and urine, were used to identify relevant biomarkers and their correlation with CKD incidence was investigated, providing a more accurate prediction of CKD diagnosis or disease aggravation.

Although AI has achieved promising results in different types of diseases such as diabetes, cancers, and cardiac diseases [22–26], its application in the field of kidney disease has been comparatively limited. The laboratory of the Massachusetts Institute of Technology established an AI prediction system for acute kidney injury. The research team collected and analyzed the electronic medical records of about 300,000 patients from the Stanford Medical Center and Beth Israel Deaconess Medical Center. AI was applied for repeated training and verification, a machine learning-based prediction model was established and showed much higher accuracy than the traditional SOFA scoring system (AUROC, 0.872 vs. 0.815) [27]. However, most of the existing AI studies on CKD have been conducted using the UCI public data. Although various algorithmic models have shown a higher diagnostic yield than traditional statistical methods, these models have large limitations due to the small data volume (<400 cases) or lack of unstructured data [28–30]. In this study, we adopted a new multimodal machine learning model, which combined MD-BERT-LGBM to identify unstructured data, which could not be realized using traditional statistics. We also discovered that the diagnostic accuracy of the five common machine learning methods was also enhanced to some degree owing to the addition of unstructured data, and among them, the accuracy of the modified XGBoost algorithm was even increased by 93.57%.

RETRACTED

Apart from urine protein, urine red blood cells and serum creatinine, we found that serum cholesterol and glycated hemoglobin were also features of high importance in this model. According to epidemiological surveys, the substantial increase in the prevalence of obesity and diabetes worldwide has made a huge difference in the incidence pattern of CKD. Metabolism-related risk factors are major drivers of CKD risk in many regions [31, 32]. Even in China, the prevalence of CKD caused by diabetes is higher than that prompted by chronic glomerulonephritis [33]. Patients with chronic nephritis and normal renal function may present with dyslipidemia, such as nephrotic syndrome, due to the disease itself. Additionally, even patients with renal insufficiency and few urinary proteins also suffer from lipoprotein metabolism disorders, dyslipidemia, and atherosclerosis due to weakening renal function [34, 35]. Uncontrolled hyperglycemia and hyperlipidemia increase the risk of cardiovascular disease and accelerate the progression of CKD to advanced stages, regardless of whether CKD is caused by diabetes or hyperlipidemia [36].

This study has several limitations to highlight. Because of the “black box” characteristics of AI algorithms, the importance score of each feature cannot serve as the correlation coefficient for the feature and the incidence of CKD, nor can a certain value be used as the cutoff point of importance score by referring to traditional statistical methods, which may lead to ignorance of other influencing factors with lower scores. Each feature cannot be independently considered to predict the incidence of CKD because their relationship is often intricate. Therefore, there are some difficulties in the clinical interpretation of the significance of each feature data. Besides, the accuracy of AI algorithms is closely related to the amount of data. Thus, another important limitation of this study is the single-center nature of this study. Therefore, these recently obtained findings should be further validated in prospective multicenter databases with multiethnic populations.

RETRACTED

## 5. Conclusion

The proposed AI prediction model could be a promising tool for the early assessment of CKD compared to traditional single-factor diagnostic methods. After further validation, if this model retains its clinical significance as demonstrated in this study, it could allow early patient referral to nephrologists for timely standardized management, thus delaying or even preventing the progression of CKD.

## Figures and Tables

**Figure 1:** Receiver operating characteristic curves of the different models. SVM, support vector machine, RF: random forest, NB, Naive Bayes, LR, Logistic regression model.

**Table 1:** Comparison of clinical data between the CKD and non-CKD groups.

Features	CKD group	Non-CKD group	Statistics	*P* value
Age (year)	63.87 ± 19.84	50.22 ± 20.45	*t* = −18.699	<0.001
Gender (male/female)	681/582	1031/917	*χ* ^2^ = 0.304	0.582
White blood cell count (^*∗*^10 ^ 9/L)	24.92 ± 0.41	24.88 ± 0.39	*t* = −2.571	0.010
Lymphocytes/monocytes	4.0 (2.9, 5.7)	4.0 (2.5, 5.5)	*Z* = −3.744	<0.001
Hemoglobin (g/L)	127.39 ± 20.24	128.21 ± 19.97	*t* = 1.137	0.256
Platelet count (^*∗*^10 ^ 9/L)	28.23 ± 0.41	28.36 ± 0.41	*t* = 8.774	<0.001
Urine glucose (positive (%))	99 (9.04%)	111 (6.09%)	*χ* ^2^ = 8.927	0.003
Urine white blood cells (positive (%))	316 (28.67%)	342 (18.62%)	*χ* ^2^ = 40.100	<0.001
Urinary occult blood (positive (%))	148 (13.52%)	181 (9.93%)	*χ* ^2^ = 8.511	0.004
Urine white blood cells (cells/*μ*L)	6 (2.22)	5 (2.14)	*Z* = −3.963	<0.001
Urine red blood cells (cells/*μ*L)	7 (4.14)	5 (3.11)	*Z* = −6.613	<0.001
Blood potassium (mmol/L)	4.00 ± 0.45	3.96 ± 0.38	*t* = −2.625	0.009
Blood sodium (mmol/L)	140.77 ± 3.67	140.66 ± 3.01	*t* = −0.820	0.412
Total cholesterol (mmol/L)	4.78 ± 1.31	4.61 ± 1.21	*t* = −3.475	0.001
Triglyceride (mmol/L)	1.30 (0.90, 2.05)	1.22 (0.87, 1.82)	*Z* = −2.764	0.006
Low-density lipoprotein (mmol/L)	2.68 ± 0.95	2.72 ± 0.84	*t* = 1.350	0.177
Total bilirubin (*μ*mol/L)	11.00 (8.20, 15.10)	11.35 (8.40, 15.40)	*Z* = −1.396	0.163
Direct bilirubin (*μ*mol/L)	3.3 (2.3, 4.9)	2.9 (2.0, 4.2)	*Z* = −6.995	<0.001
Alanine aminotransferase (mmol/L)	17.0 (12.0, 25.0)	17.0 (12.0, 26.5)	*Z* = −1.252	0.211
Fasting blood glucose (mmol/L)	5.52 (4.86, 6.70)	5.05 (4.56, 5.71)	*Z* = −11.647	<0.001
Blood urea nitrogen (mmol/L)	5.26 ± 1.97	4.77 ± 1.79	*t* = −7.015	<0.001
Serum creatinine (*μ*mol/L)	70.79 ± 18.11	62.19 ± 16.38	*t* = −13.351	<0.001
Blood uric acid (*μ*mol/L)	302.18 ± 104.63	292.58 ± 94.92	*t* = −2.580	0.010
Albumin (g/L)	41.08 ± 4.95	40.67 ± 5.23	*t* = −2.158	0.031
Globulin (g/L)	26.76 ± 5.31	26.10 ± 4.61	*t* = −3.541	<0.001
Thrombin time (s)	17.27 ± 1.91	16.64 ± 2.94	*t* = −3.561	<0.001
International normalized ratio	1.03 ± 0.24	1.00 ± 0.12	*t* = −3.828	<0.001
Fibrinogen (g/L)	3.11 ± 1.13	3.09 ± 1.12	*t* = −0.244	0.807

Note: lymphocyte/monocyte, ratio of peripheral blood lymphocyte count to monocyte count.

RETRACTED

**Table 2:** Correlation analysis between the incidence of CKD and laboratory test indicators.

Features	*r*	*P* value
^*∗*^ Neutrophils (%)	0.122	<0.001
^*∗*^ White blood cell count (^*∗*^10^9/L)	0.053	0.003
^*∗*^ Red blood cell distribution width (%)	0.102	<0.001
Red blood cell count (^*∗*^10^12/L)	−0.075	<0.001
^*∗*^ Platelet count (^*∗*^10^9/L)	−0.185	<0.001
Platelet distribution width (%)	−0.077	<0.001
^*∗*^ Urine red blood cells (cells/*μ*L)	0.129	<0.001
Urinary occult blood (positive/negative)	0.053	0.004
^*∗*^ Urine white blood cells (positive/negative)	0.117	<0.001
Urine white blood cells (cells/*μ*L)	0.077	<0.001
^*∗*^ Thrombin time (s)	0.160	<0.001
Prothrombin time (s)	0.111	<0.001
International normalized ratio	0.026	0.167
^*∗*^ Blood urea nitrogen (mmol/L)	0.136	<0.001
^*∗*^ Serum creatinine (*μ*mol/L)	0.226	<0.001
^*∗*^ Blood uric acid (*μ*mol/L)	0.047	0.008
^*∗*^ Globulin (g/L)	0.054	0.002
Albumin (g/L)	0.026	0.141

Note: ^*∗*^refers to the feature retained after deletion of features with similar clinical significance according to the size of the correlation coefficient.

**Table 3:** Ranking of the top 15 XG Boost model features.

Features	*P* value
Protein	0.220
Urine red blood cells	0.209
Age	0.050
Serum-creatinine	0.032
Gender	0.017
Albumin-creatinine ratio	0.015
Leukocyte	0.013
Erythrocyte	0.013
Platelet distribution width	0.009
High-sensitivity C-reactive protein	0.008
Hemoglobin	0.008
Hemoglobin A1c	0.008
Platelet	0.008
Albumin	0.007
Potassium	0.007

**Table 4:** Prediction performance of the different models.

Model	Indicator				Indication with MD-BERT-LGBM			
	Accuracy	Precision	Recall	AUC	Accuracy	Precision	Recall	AUC
XGBoost	0.9088	0.9175	0.8244	0.9549	0.9357	0.9425	0.8782	0.9719
SVM	0.8048	0.8330	0.5828	0.8705	0.7992	0.8392	0.5575	0.8704
NB	0.7811	0.8326	0.4973	0.8460	0.8086	0.8670	0.5556	0.7693
RF	0.9020	0.9318	0.7905	0.9519	0.9108	0.9550	0.7927	0.9716
LR	0.8276	0.7868	0.7225	0.8903	0.8489	0.8187	0.7551	0.9045

SVM, support vector machine, RF, random forest, NB, Naïve Bayes, LR, logistic regression model.

RETRACTED

## Data Availability

The data used to support the findings of this study are available from the corresponding author upon request.
